The article "Identification of the Sites of Tau Hyperphosphorylation and Activation of Tau Kinases in Synucleinopathies and Alzheimer’s Diseases" was retracted in 2025. Reasons: original data or images not available; unreliable results or conclusions; concerns about the images.

# Identification of the Sites of Tau Hyperphosphorylation and Activation of Tau Kinases in Synucleinopathies and Alzheimer’s Diseases

**DOI:** 10.1371/journal.pone.0075025

**Published:** 2013-09-20

**Authors:** Valeriy Duka, Jae-Hoon Lee, Joel Credle, Jonathan Wills, Adam Oaks, Ciaran Smolinsky, Ketul Shah, Deborah C. Mash, Eliezer Masliah, Anita Sidhu

**Affiliations:** 1 Department of Biochemistry and Molecular & Cellular Biology, Georgetown University Medical Center, Washington, District of Columbia, United States of America; 2 Department of Neurology and Molecular and Cellular Pharmacology, Miller School of Medicine, University of Miami, Miami, Florida, United States of America; 3 Department of Neuroscience, University of California San Diego, La Jolla, California, United States of America; Oregon Health & Science University, United States of America

## Abstract

**Objective:**

Most neurodegenerative diseases contain hyperphosphorylated Tau [p-Tau]. We examined for the first time epitopes at which Tau is hyperphosphorylated in Parkinson’s disease, dementia with Lewy bodies and Alzheimer’s disease, and also select Tau kinases.

**Methods:**

Postmortem frontal cortex from Parkinson’s disease, dementia with Lewy bodies, Alzheimer’s disease and striata from Parkinson’s disease, were analyzed by immunoblots using commercially available antibodies against 20 different phospho-epitopes of Tau. Major Tau kinases were also screened. Results in diseased tissues were compared to nondiseased controls.

**Results:**

In Alzheimer’s disease, Tau was hyperphosphorylated at all the 20 epitopes of p-Tau. In dementia with Lewy bodies, p-Tau formation occurred at 6 sites sharing 30% overlap with Alzheimer’s disease, while in Parkinson’s frontal cortex, an area which does not degenerate, Tau hyperphosphorylation was seen at just 3 epitopes, indicating 15% overlap with Alzheimer’s disease. In Parkinson’s disease striatum, an area which undergoes considerable neurodegeneration, Tau was hyperphosphorylated at 10 epitopes, sharing 50% overlap with Alzheimer’s disease. Between frontal cortex of Parkinson’s disease and dementia with Lewy bodies, there were only two p-Tau epitopes in common. In striata of Parkinson’s disease, there were 3 clusters of Tau hyperphosphorylated at 3 contiguous sites, while two such clusters were detected in dementia with Lewy bodies; such clusters disrupt axonal transport of mitochondria, cause microtubule remodeling and result in cell death. p-GSK-3β, a major Tau kinase, was activated in all brain regions examined, except in dementia with Lewy bodies. Activation of other Tau kinases was seen in all brain regions, with no clear pattern of activation.

**Interpretation:**

Our studies suggest that the three neurodegenerative diseases each have a signature-specific profile of p-Tau formation which may be useful in understanding the genesis of the diseases and for the development of a panel of specific biomarkers.

## Introduction

Alzheimer’s and Parkinson’s disease [PD] are the two most common neurodegenerative diseases of the elderly, while dementia with Lewy bodies [DLB] is the second-most common form of dementia after Alzheimer’s disease [AD]. AD is characterized by extraneuronal plaques comprised of β-amyloid [A-β], and intraneuronal aggregates and tangles of the microtubule [MT] associated protein, Tau, abnormally hyperphosphorylated at numerous toxic epitopes [1-3]. The synucleinopathies, PD and DLB, are characterized by intraneuronal aggregates of a different amyloidogenic protein, α-synuclein [α-Syn], which accumulates into Lewy bodies and Lewy neurites [4,5], in dopaminergic neurons of the mid-brain of PD and frontal cortex [FC] of DLB, respectively. While abnormal hyperphosphorylation of Tau has been extensively studied in the context of AD and related tauopathies, virtually nothing is known about p-Tau in degenerative diseases such as PD and DLB. This is likely because p-Tau is generally hyperphosphorylated at fewer sites in non-tauopathic diseases, and therefore has not been considered to be central to the disease process. In addition, it has long been assumed that much of the pathology was due to the amyloidogenic proteins. However, this view is increasingly challenged [6,7], since neurodegenerative diseases show increasing similarities in pathologies in terms of axonal transport disruption, protein aggregation, synapse loss and accumulation of protein aggregates, including p-Tau. Even in diseases that contain only a few p-Tau sites, it was found that hyperphosphorylation at just 3 p-Tau epitopes can cause neurodegeneration [8,9].

While basal levels of phosphorylated Tau promotes axonal stability, enabling synaptic plasticity and axonal transport of organelles to and from cell bodies to nerve terminals [10], its hyperphosphorylation at certain epitopes in the adult brain is pathological and specifically related to degeneration, cognitive impairment and dementias [11]. Hyperphosphorylation of Tau causes the protein to detach from axons, inducing microtubule remodeling and compromising axonal transport [8-11]. In familial and sporadic tauopathies [11], there is clear evidence showing that Tau pathology alone can cause neurodegeneration.

The state of Tau hyperphosphorylation in DLB is unknown and there have been only very limited studies on p-Tau in PD. Tau was found to be hyperphosphorylated at Ser396 in FC synaptosomes in postmortem PD tissues [12]. Using a small number number of antibodies, we found Tau to be hyperphosphorylated at Ser202, Ser262 and Ser396/404 in PD striata [13]. Limited tauopathy in different non-degenerating brain regions in the α-Syn transgenic mouse model of PD was also seen [14]. In cellular and animal models of PD, our past studies demonstrate that both α-Syn and reactive oxygen species [ROS] are essential for p-Tau formation [15-21] and in the absence of either component p-Tau is not induced [15-17,21]. An additional feature of p-Tau formation in PD is GSK-3β, a major Tau kinase capable of hyperphosphorylating Tau at a majority of its sites, after it is activated by autophosphorylation at Tyr216 [17,18]. Most interestingly, we found in animal models of PD, that p-GSK-3β-Tyr216 expression was restricted to midbrain and striatum, areas which contain dopamine neurons, have high levels of α-Syn, produce ROS and which degenerate in this disease [14]. Inhibition of p-GSK-3β-Tyr216 prevented, and even reversed p-Tau formation [17,18]. Indeed, addition of lithium or TDZD-8 [a highly selective inhibitor of p-GSK-3β-Tyr216] when added to dying neuronal cells 36 h after initiation of toxicity with ROS, was sufficient to reverse cell death and aggregation of both α-Syn and p-Tau within 12 h [17]. Thus, targeting p-GSK-3β may prove to be useful in the development of novel treatments for PD.

Since virtually nothing is known about p-Tau in either PD or DLB, we sought to undertake a comprehensive analyses identifying the number of epitopes of Tau that are hyperphosphorylated in different brain regions of these diseases, while also investigating the activation of various Tau kinases. For our studies, we used postmortem FC of PD, DLB and AD, so that comparisons could be made across a single brain region among different diseases. In addition, we also examined PD striatum. Our data shows that each disease and brain region has a distinct pattern of Tau hyperphosphorylation, with a strong correlation between the number of p-Tau sites and degeneration. Moreover, different Tau kinases were found to be activated in the various diseases, with differences seen among brain regions even within the same disease. Our results have identified for the first time the state of Tau hyperphosphorylation in PD and DLB, which may be useful in not only understanding the genesis of these diseases at the molecular level, but also for the development of specific p-Tau and Tau kinase biomarkers.

## Materials and Methods

### Antibodies

All studies with animals were approved by the Georgetown University Institutional Animal Care and Use Committee (Protocol 10-076). The antibodies used in this study are listed in Table S1 in File S1, and include information of the companies the antibodies were purchased from, catalog numbers, working dilutions and target sites. To assess specificity of the 20 p-Tau antibodies used in our studies, Western blots were conducted using lysates isolated from mice striata overexpressing human Tau P301S and Tau knock out mice [see Figure S1 in File S1]. As seen from these results, all antibodies showed very high specificity against the p-Tau epitope of interest, indexed by lack of detection of any protein in the Tau knock out mouse.

### Postmortem tissue

All studies using autopsied materials were approved by the Institutional Review Board of Georgetown University. Informed consent was obtained by the Brain data banks, patient identity was not disclosed to researchers and all data was analyzed anonymously. Details of the brains [genders, age of donors and postmortem interval] used in this study are listed elsewhere [13,22,23]. Briefly, postmortem PD striata or FC [N=10] was provided by either the Sun Health Research Institute, Brain and Body Donation Program [Sun City, AZ] or from the University of Miami, Brain Endowment Bank^TM^ [Miami, FL] and included samples from PD cases without dementia and neuropathologically confirmed to be absent any AD pathology. Frontal cortex of DLB [N=6] and AD [N=10] were provided by the brain bank of University of California at San Diego [San Diego, CA]. Both DLB and AD tissues were analyzed neuropathologically and confirmed to contain cortical Lewy bodies or AD pathology, respectively. Age-matched controls subjects were evaluated by cognitive tests prior to death and were confirmed at autopsy to be free of brainstem or cortical Lewy Bodies. Control subjects had normal age-adjusted senile plaque scores and were free of neurofibrillary tangles. The postmortem interval ranged from 3-18 hours, with an average of ~9 hours. Tissues from both males and females were used, as there were no gender differences.

### Preparation of lysates and Western blot analyses

Tissues were homogenized [13] in buffer containing 10 mM Tris HCL, pH 7.4,1M NaCl, 250 mM Sucrose, 5 mM KCl, 2 mM CaCl_2_, 1 mM MgCl_2_, 1 mM dithiothreitol, 1 mM EDTA, 1 mM EGTA, 10 µg/ml each of phosphatase inhibitor cocktail [Halt Phosphatase inhibitor Cocktail; Thermo Scientific, Rockford, IL] and protease inhibitor cocktail tablets [Complete Mini, EDTA-free; Roche Diagnostics, Mannheim, Germany], and 500 µM PMSF. Sodium cholate [20% in water, wt/vol] was added to a final concentration of 2% [vol/vol] and the mixture was briefly vortexed and left on ice for 30 min, with occasional vortexing, followed by centrifugation for 45 min at 30,000 x *g* at 4 °C. This method yields superior solubility of synucleins, kinases and p-Tau proteins in a single preparation, than any other detergent and solubilization procedure we have tried [13]. Since all proteins, including α-Syn, β-amyloid and p-Tau proteins were predominantly [>95%] found in the supernatant fractions and not in pellets, only supernatant fractions were analyzed in this study. Supernatants were collected and protein concentrations were measured using the Lowry assay after diluting samples with dilution buffer [10 mM Tris HCL, pH 7.4, 250 mM Sucrose, 5 mM KCl, 2 mM CaCl2, 1 mM MgCl2, 1 mM dithiothreitol, 1 mM EDTA, 1 mM EGTA, 10 µg/ml each of phosphatase inhibitor cocktail and protease inhibitor cocktail tablets, and 500 µM PMSF] to a final concentration of 0.2% of sodium cholate. The clear supernatants were mixed with Laemmli buffer [1: 1 vol/vol] and heated in boiling water for 5 min, and Western blot analyses were performed [13]. All phospho-proteins were calculated relative to their non-phosphorylated proteins and were normalized to either actin or GAPDH.

### Immunohistochemistry

Five micron sections from formalin-fixed paraffin-embedded tissues were de-paraffinized with xylenes and rehydrated through a graded alcohol series. Heat induced epitope retrieval [HIER] was performed by immersing the tissue sections at 98°C for 20 minutes in 10 mM citrate buffer [pH 6.0] with 0.05% Tween. Immunohistochemical staining was performed using a horseradish peroxidase labeled polymer from Dako [K4003, K4000] according to manufacturer’s instructions. Briefly, slides were treated with 3% hydrogen peroxide and 10% normal goat serum for 10 minutes each, and exposed to 1:500 dilutions of primary antibodies for 1hr at room temperature. Slides were exposed to anti-mouse labeled HRP for 30 min and DAB chromagen [Dako] for 5 minutes. Slides were counterstained with Hematoxylin [Fisher, Harris Modified Hematoxylin] at a 1:17 dilution for 2 minutes at room temperature, blued in 1% ammonium hydroxide for 1 minute at room temperature, dehydrated, and mounted with Acrymount. Sections with the omitted primary antibody served as negative controls.

### Statistical analysis

Results were expressed as mean ± S.E.M. and statistically analyzed by the Student’s t test between two groups and analysis of variance among multiple groups. Statistical significance was accepted at the [*P*<0.05] level.

## Results

### Identification of sites of hyperphosphorylation of Tau

We have previously shown elevated levels of p-Tau, hyperphosphorylated at Ser202, Ser262 and Ser396/404 in postmortem striata of patients with PD [13]. In postmortem frontal cortex of PD patients, however, we failed to detect these sites [13]. However, an independent study reported the presence of Ser396 in FC synaptosomes [12]. Using Western blots and all p-Tau antibodies that are commercially available, we conducted a thorough investigation of 20 hyperphosphorylated epitopes of Tau in postmortem PD FC and striata, and in FC of DLB and AD. In human tissues, there is large variation in results from sample to sample. To show these variations, scatter plots were created to show deviations we encountered in each of our control and diseased samples.

In PD FC, significantly increased [by ~150, 100 and 100%, respectively] hyperphosphorylation of Tau occurred at just three sites, Ser238, Ser356 and Ser413 [Figure 1A and Table S2 in File S1]. Consistent with our previous studies, we once again failed to detect any significant phosphorylation at Ser202, Ser262 and Ser396/404 [13]. The presence of only 3 hyperphosphorylated in PD FC indicates 15% overlap in homology in with AD FC.

**Figure 1:** Identification of Tau phosphorylation sites in postmortem human FC from PD, DLB AD and PD striata. Western blot analyses of p-Tau levels were conducted using specific p-Tau antibodies as described in Materials [see Table S1 in File S1]. [A] postmortem FC of human PD cases [N = 7-9] and non-diseased controls [N = 7]; [B] FC from human DLB cases [N = 7-10] and non-diseased controls [N = 7-10]; [C] postmortem FC from human AD cases [N = 5-6] and non-diseased controls [N = 4-6], [D] postmortem striata from human PD cases [N = 7-9] and non-diseased controls [N = 7-10]; Summary of quantitation for opticzal density [OD] of each p-Tau site relative to total Tau is presented as percent of age-matched control. Due to large variation in human tissues, scatter plots were drawn to show variations within each individual control sample [blue squares] or diseased sample [red circles]. Bars show group means ± SEM. Data for each p-Tau site were analyzed by t-test for difference from the control group [*p<0.05].

In DLB FC, significant Tau hyperphosphorylation was seen at 7 sites: Thr212, Ser214, Thr217, Thr231, Ser238, Ser396/404 and Ser422 [Figure 1B and Table S2 in File S1], indicating 35% overlap in homology with AD. Compared to PD FC, there were only two sites common to DLB FC, Ser238 and Ser 396/404, suggesting an overlap of 10% of p-Tau epitopes between these two diseases. Interestingly, in DLB, levels of Thr231 were decreased compared to controls, which were not observed in other diseases or for any other epitope. In DLB FC, there appears to be 2 clusters of 3 contiguous sites of p-Tau: Thr212/Ser214/Thr217 and Ser396/404/Ser422. The presence of such clusters may have important roles in the degenerative process in this disease, and previous studies have found that a single such contiguous cluster was sufficient to disrupt axonal transport of mitochondria, due to microtubule remodeling, resulting in cell death [8]. Although DLB FC appears to contain only a few hyperphosphorylated sites, the relatively high levels of p-Tau may have an important role in the dementia associated with this disease.

When we conducted parallel studies in postmortem AD FC, all of the 20 epitopes examined showed significantly increased hyperphosphorylation of Tau [Figure 1C and Table S2 in File S1], consistent with earlier findings [1,2], that Tau in PD is hyperphosphorylated at all these 20 epitopes.

We next examined PD striatum, since this is a region known to degenerate in PD, and is likely to have the largest number of p-Tau sites. Indeed, significantly [p <0.05] increased levels of p-Tau were found to be hyperphosphorylated at 10 epitopes: Ser202, Thr205, Thr212, Ser235, Ser262, Ser356, Ser396/404, Ser409, Ser413 and Ser422, compared to controls [Figure 1D and Table S2 in File S1]. There were no significant [p>0.05] increases in hyperphosphorylation at the rest of the p-Tau sites examined [Figure 1D]. Since 10 out of 20 sites tested were similar to AD [see Figure 1C], the overlap in p-Tau homology between PD striatum and AD FC is 50%. Between PD striatum and PD FC, only Ser356 and Ser413 were common to both these brain regions within the same disease, while PD striatum and DLB FC shared 3 epitopes in common [Thr212, Ser396/404 and Ser422]. Most interestingly, in PD striatum, there appeared to be 3 clusters of contiguous sets of 3 p-Taus: Ser202/Thr205/Thr212, Ser356/Ser396/Ser404 and Ser409/Ser413/Ser422. Each of these clusters, either separately or in synergy have the potential to contribute to the neurodegeneration of PD striatum.

### Analyses of synucleins

A common feature of neurodegenerative diseases [such as PD, prion disease, AD, Huntington’s disease and DLB] is the presence of elevated levels of aggregated amyloidogenic proteins [α-Syn, prion, β-amyloid, huntingtin or α-Syn, respectively] [24]; upon aggregation, α-Syn which is normally present in a disordered soluble form, becomes amyloidogenic. When the levels of the members of the Syn family, α-, β- and γ-Syn, were analyzed in FC of PD [Figure 2A] and DLB [Figure 2B], significant increases were seen in the levels of α-Syn and γ-Syn. However there were no significant changes in levels of β-Syn in either PD or DLB FC. In AD, significant increases were seen only for α-Syn [Figure 2C], while levels of β-amyloid were increased 15-fold [Figure 2C]; β-amyloid was absent in both PD and DLB [data not shown]. In PD striatum, increased levels of all 3 synucleins were observed [Figure 2D]. Increases in β-Syn have been reported to counter the toxic effects of α-Syn [25,26] and lack of its activation in PD FC, DLB and AD may suggest that the effects of α-Syn in these diseases may be more noxious. Further, γ-Syn has been shown to participate in neurodegeneration [27], and increases in this protein in both PD and DLB suggest that γ-Syn may synergize with α-Syn toxicity in synucleinopathies.

**Figure 2:** Expression of synuclein proteins in FC of PD, DLB, AD and PD striata. [A] Postmortem PD FC from [N = 7-9] diseased and [N = 7] non-diseased controls, [B] FC from DLB cases [N = 7-10] and non-diseased controls [N = 7-10], [C] FC from AD cases [N = 5-6] and non-diseased controls [N = 4-6], and [D] Striata from PD cases [N = 7-9] and non-diseased controls [N = 7-10]; were analyzed using immunoblots for expression of α-Syn, β-Syn, and γ-Syn, using antibodies listed in Table S1 in File S1. OD of each protein relative to GAPDH is presented as percent of corresponding non-diseased control cases [mean ± SEM]. Data for each Syn protein were analyzed by t-test for difference from corresponding control group [*p<0.05; **p<0.01].

### Activation of Tau kinases

The epitopes at which Tau is hyperphosphorylated is dependent on specific Tau kinases, with most kinases having considerable overlapping abilities to phosphorylate the various epitopes of Tau [1,2]. In PD FC, there was significant activation of p-GSK-3β [phosphorylated at Tyr216 and representing the active form of the kinase], p-p38MAPK and protein kinase A [PKA], with no changes in either p-ERK [phospho-extracellular signal-regulated kinase], p-JNK [phospho-c-Jun N-terminal kinase] or in cdk5, nor in any of its activator proteins, p35 or p25 [Figure 3A]. p-GSK-3β has emerged as a major and important Tau kinase, since it can hyperphosphorylate Tau at the majority of its ~45 epitopes [1,2].

**Figure 3:** Identification of Tau kinases activated in FC of PD, DLB, AD and PD striata. **[A]**. FC from PD and non-diseased controls, [B] FC from DLB cases and non-diseased controls, [C] FC from AD cases and non-diseased controls, and [D] Postmortem striata from PD cases and non-diseased controls, were probed using immunoblots for expression of the various Tau kinases, using antibodies listed in Table S1 in File S1. N values for all samples were as listed in legend to Figure 1. Activating phosphorylations of p-GSK-3β, p-ERK, p-JNK, and p-p38 were probed in parallel with phospho-specific antibodies [see Table S1 in File S1]. OD was analyzed as total kinase relative to GAPDH [p35, p25, cdk5, and PKA] or as phosphorylated kinase relative to total kinase [GSK-3β. JNK, p39MAPK and ERK] and are presented as percent of corresponding control cases [mean ± SEM]. Data for each kinase were analyzed by t-test for difference from corresponding control group [*p<0.05; **p<0.01].

In DLB FC [Figure 3B], there were significant increases in p-ERK, p-JNK and p-p38MAPK, along with increases cdk5 and its activator proteins [p35 and p25]. There were also no increases in p-GSK-3β or PKA levels in DLB [Figure 3C]. AD FC, increased levels of p-GSK-3β, p-p38MAPK, PKA and cdk5 along with its activators, p35 and p25 proteins, were seen [Figure 3C]. For p-JNK, reduced levels of this kinase were observed, but the decrease was not significant. There were also no significant changes in levels of either p-JNK or p-ERK in AD frontal cortex.

In PD striatum [Figure 3D], robust increases were seen in the majority of the Tau kinases: p-GSK-3β, p-JNK, p-p38MAPK, and cdk5, including increases in its p35 and p25 activator proteins and in PKA. However, we did not find any significant changes in p-ERK levels. The activation of cdk5 was previously reported in the MPTP mouse model of PD, where elevations in this kinase were noted immediately after initiation of treatment with the neurotoxin, abating toward the end of the treatment, suggesting that cdk5 may be involved in the early stages of the disease pathology [28]. The increases in PKA are also consistent with earlier studies in *in vitro* models of PD, where PKA activation was seen in cell-free systems [29] as well as in cells [30]. Most interesting is the fact that although nearly the same number of kinases was activated in PD FC and in PD striatum, there was a large difference in the number of Tau sites that were hyperphosphorylated, 3 versus 10, respectively. While it can be argued that this difference may be due to the activation of cdk5 in PD striatum, we believe that this difference is likely due to the additional presence of ROS in the degenerating striatum. As mentioned earlier, a key component in the α-Syn-mediated hyperphosphorylation of Tau is highly dependent on the presence of ROS [17,21], which in the striatum could arise due to metabolism of DA or dysfunctional mitochondria. Moreover, in PD mouse models, we have previously observed that brain regions which do not contain high levels of ROS, such as frontal cortex, cerebellum and hippocampus, there is also much fewer hyperphosphprylation of Tau in these regions [14].

### Immunohistochemistry of p-Tau [Ser396/404] and α-Syn in PD, DLB and AD brains

We examined α-Syn and p-Tau [pSer396/404] in these diseases by immunohistochemistry. Due to lack of PD frontal cortex slices, PD striata was used in these studies. In PD striata, α-Syn was present as aggregates which accumulated in large intraneuronal Lewy bodies and in Lewy neurites [Figure 4A]. A similar pattern of immunostaining was also seen in DLB [Figure 4A], where lower levels of α-Syn was accumulated in Lewy bodies, and which, moreover, were smaller in size relative to PD. In AD, Lewy bodies and Lewy neurites were notably absent, although low levels of α-Syn aggregates were observed throughout the neuron [Figure 4A]. Intracellular immunostaining of p-Tau [Ser396/404] showed this protein to be present as aggregates throughout the cell bodies of neurons in PD and AD [Figure 4B]. Furthermore, distinct extraneuronal tangles of p-Tau were observed in AD, but not in PD or DLB. There were only very low levels of Ser396/404 seen in DLB, consistent with low levels of these epitopes detected by Western blots.

**Figure 4:** Immunohistochemical analyses of α-Syn and p-Tau. IHC of paraffin embedded tissue from AD FC, PD substantia nigra and DLB FC with appropriate aged matched non-diseased controls, were conducted as described in Methods of File S1. [A] Analysis of α-Syn associated pathology in PD [uppermost horizontal panel], DLB [middle horizontal panel] and AD [lower horizontal panel] comparing age matched control tissue [left vertical panel] with diseased tissue [middle and right-magnified vertical panels]. Lewy bodies increased in intensity and density as follows: PD > DLB > AZ. * denotes Lewy bodies and were present only in PD and DLB tissues. [B] Analysis of p-Ser396/404 associated pathology in AD [uppermost horizontal panel], PD substantia nigra [middle horizontal panel] and DLB [bottom horizontal panel], compared age matched control tissue [left vertical panel] with diseased tissue [middle and right-magnified]. * Aggregates, ** Tangles.

## Discussion

A schematic of our findings of p-Tau in the various diseases are displayed in Figure 5, where the position of these hyperphosphorylated sites on the Tau can be easily seen and compared.

**Figure 5:** Schematic of Tau phosphorylation in PD, DLB, and AD. Full length Tau [2N4R] contains ~45 known Thr/Ser sites known to be hyperphosphorylated in AD. These sites are spread throughout several regions of Tau, including the E2/E3 domains, the proline-rich domain, the MT-binding domain, and the C-terminal of the Tau protein. Phosphorylation at 20 sites [Table S1 in File S1] was analyzed in PD striata [bottom] and DLB FC [top]. Sites with elevated phosphorylation are indicated in red, while sites where phosphorylation was similar to controls are indicated in blue. A decrease in phosphorylation at T231 was identified in DLB tissues [green]. Sites in orange represent hyperphosphorylated sites present in DLB FC. Sites in black denote epitopes not tested in PD or DLB or AC. All sites shown, regardless of color, are hyperphosphorylated in AD.

Although much interest has been focused on the role of amyloidogenic proteins in neurodegenerative diseases, recent attention has shifted to p-Tau, as this protein rather than the amyloid proteins, can more adequately account for loss of nerve terminals, due to their effects on microtubular remodeling and axonal transport deficiencies. While much attention has classically been devoted to analyzing p-Tau in AD and other tauopathies, the role of p-Tau in non-AD states has been largely neglected, partly due to a broad misconception that Tau toxicity only occurs when a large number of epitopes are hyperphosphorylated. However, this notion has been increasingly challenged, as more reports suggest that formation of p-Tau may be a common denominator in neurodegenerative events [6,7]. In particular, two recent reports have shown that hyperphosphorylation of Tau at just 3 contiguous sites, Ser199/Ser202/Thr205 [8], or at semi-contiguous sites, Thr212/Thr231/Ser262 [9], was sufficient to cause microtubule remodeling and instability, diminished mitochondrial transport, cell death and neurodegeneration.

In PD striatum, we found at least 3 clusters containing 3 contiguous p-Tau sites: Ser202/Thr205/Thr212, Ser262/Ser356/Ser396 and Ser404/Ser409/Ser422 [Figure 5]. Some or all of these clusters may independently or synergistically act to trigger microtubule changes, loss of axonal transport, mitochondrial deficits and death of nerve terminals, features that are all too common in PD. In DLB FC, two clusters of 3 contiguous sites were identified, Thr212/Ser214/Thr217 and Ser396/Ser404.Ser42. Interestingly, in PD FC, the 3 epitopes of p-Tau, Ser238, Ser356 and Ser413 occur far apart from one another, which may explain why the FC in PD does not degenerate. However, the presence of these p-Tau sites may contribute to the FC-dependent cognitive changes associated with PD. It should be noted that although Tau can be hyperphosphorylated at ~45 epitopes, very few studies have been conducted in AD on the specific roles of each of these sites in neurodegeneration, or even clusters of sites. Thus, the function and molecular consequences of the majority of p-Tau are not known in either AD, which is the best studied disease with regard to PD, or in other tauopathies.

Tau hyperphosphorylation is mediated by several kinases, many of which show large overlap in their ability to phosphorylate Tau at the same epitopes, making it hard to assign phosphorylation of a specific site to a particular kinase, or vice versa. Of the Tau kinases, p-GSK-3β has emerged as the single most important kinase, as it can hyperphosphorylate Tau at the majority of its epitopes [1,2]. A l12 month clinical trial using Li to block GSK-3β in AD significantly decreased CSF concentrations of p-Tau (P = 0.03) with improvement in cognitive attention tasks [31]. Our earlier studies have identified p-GSK-3β as a major kinase in cellular and animal models of PD [15-17], and blockade of this kinase was sufficient to abolish and reverse p-Tau formation and α-Syn aggregation [15-17]. Thus, targeting this kinase may hold promise in the development of novel therapies for neurodegenerative diseases.

Although cdk5 [24,28] is an important kinase in AD, it may not have a role in PC of PD or DLB due to lack of activation, whereas in PD striatum, this kinase may be an important participant. The MAPK family of kinases is also known to abnormally phosphorylate Tau at overlapping sites [32-35]. In FC of both PD and DLB, we observed upregulation of p-JNK, with increases also seen in PD striatum, but not in AD. Interestingly, p-p38MAPK levels were increased across all diseases and tissues, while p-ERK was unchanged. It is likely that the overlap in p-Tau epitopes [Thr212, Ser396/404 and Ser422] seen in PD striatum and DLB FC is due to p-JNK and/or p-p38MAPK, since p-p38MAPK can phosphorylate Tau at Ser46, Thr181, Ser202, Thr205, Thr212, Thr217, Thr231, Ser235, Ser356, Ser396/Ser404, while p-JNK phosphorylates Tau at Thr212, Thr217, Ser396/404 and Ser422 [1]. These findings support our contention that the overlap in p-Tau epitopes between PD striatum and DLB occurs through a common activation of these two MAPKs.

In a M17 cell model of PD [30], activation of PKA in an α-Syn-dependent manner leading to Tau phosphorylation has been described, but the findings were not confirmed in human diseased tissues. We found an upregulation of PKA in PD striatum and FC, and AD, but not DLB. PKA phosphorylates Tau at Thr181, Ser214, Thr217, Thr231, Ser262 and Ser409, as well as Ser422 [1], and PKA-dependent phosphorylations of Tau at Thr231 precede or are coincident with the initial appearance of filamentous aggregates of Tau [35]. Although some of the PKA-dependent epitopes are not found in PD [Thr181, Ser214, Thr217, Thr231], other putative PKA sites do exist [Ser262, Ser409 and Ser422] and PKA well may be the kinase involved in this process. In DLB, whereas phosphorylation is seen at Ser214, Thr217, Thr231 and Ser409, lack of phosphorylation at Thr181, Ser262 and Ser409, together with no changes in PKA, indicates a lack of participation of this kinase in DLB.

The list of p-Tau epitopes and Tau kinases presented in this paper is by no means complete or all encompassing, since other sites of p-Tau are yet to be identified, some of which may be unique to the disease. In order to identify all the p-Tau sites, mass spectroscopy will need to be conducted [36], which is by no means a trivial undertaking. Still, our studies are a first step in cataloguing and documenting the different p-Tau epitopes and Tau kinases present in PD FC and striatum, and in DLB FC. Importantly, our results suggest that different neurodegenerative diseases have distinct signature-specific patterns of Tau hyperphosphorylation and kinase activation. This information may be important not only for understanding the differences between these diseases at the cellular level, but also for understanding associated molecular pathways. Most importantly, our studies hold special value for the development of unique biomarkers, comprising of p-Tau epitopes and activated kinases that may be useful in identifying early disease signatures. Finally, targeting specific p-Tau sites and Tau kinases with small molecule inhibitors or through passive immunization may be useful for development of novel, individualized therapies to slow, or even reverse, the progression of a disease. In this regard, a recent study has shown that Tau immunotherapy targeting p-Ser422 in the THY-Tau22 transgenic mouse model of AD, significantly improved cognitive performance in the Y maze test [37]. Similar approaches targeting selective p-Tau in PD and DLB may represent novel and unique approaches in the treatment of these diseases.

## Supporting Information

File S1 **Materials and methods, Tables S1 and S2, Figure S1.**
(DOC)

## References

[1] HangerDP, AndertonBH, NobleW (2009) Tau phosphorylation: the therapeutic challenge for neurodegenerative disease. Trends Mol Med 15: 112-119. doi:10.1016/j.molmed.2009.01.003. PubMed: 19246243.1924624310.1016/j.molmed.2009.01.003

[2] IqbalK, LiuF, GongCX, Grundke-IqbalI (2010) Tau in Alzheimer disease and related tauopathies. Curr Alzheimer Res 7(8): 656-664.2067807410.2174/156720510793611592PMC3090074

[3] LippensG, AmniaiL, WieruszeskiJM, SillenA, LeroyA et al. (2012) Towards understanding the phosphorylation code of tau. Biochem Soc Trans 40(4): 698-703. doi:10.1042/BST20120050. PubMed: 22817719. Review.2281771910.1042/BST20120050

[4] GoedertM, SpillantiniMG (1998) Lewy body diseases and multiple system atrophy as alpha-synucleinopathies. Mol Psychiatry 3: 462-465. doi:10.1038/sj.mp.4000458. PubMed: 9857966.985796610.1038/sj.mp.4000458

[5] DauerW, PrzedborskiS (2003) Parkinson’s disease: mechanisms and models. Neuron 39: 889-909. doi:10.1016/S0896-6273(03)00568-3. PubMed: 12971891.1297189110.1016/s0896-6273(03)00568-3

[6] JellingerKA (2012) Interaction between pathogenic proteins in neurodegenerative disorders. J Cell Mol Med 16(6): 1166-1183. doi:10.1111/j.1582-4934.2011.01507.x. PubMed: 22176890.2217689010.1111/j.1582-4934.2011.01507.xPMC3823071

[7] GilleyJ, AdalbertR, ColemanMP (2011) Modelling early responses to neurodegenerative mutations in mice. Biochem Soc Trans 39(4): 933-938. doi:10.1042/BST0390933. PubMed: 21787326.2178732610.1042/BST0390933

[8] ShahpasandK (2012) Regulation of mitochondrial transport and inter-microtubule spacing by tau phosphorylation at the sites hyperphosphorylated in Alzheimer's disease . J Neurosci 32(7): 2430-2441. doi:10.1523/JNEUROSCI.5927-11.2012. PubMed: 22396417.2239641710.1523/JNEUROSCI.5927-11.2012PMC6621814

[9] AlonsoAD, Di ClericoJ, LiB, CorboCP, AlanizME et al. (2010) Phosphorylation of tau at Thr212, Thr231, and Ser262 combined causes neurodegeneration. J Biol Chem 285: 30851-30860. doi:10.1074/jbc.M110.110957. PubMed: 20663882.2066388210.1074/jbc.M110.110957PMC2945578

[10] LovestoneS, ReynoldsCH (1997) The phosphorylation of tau: a critical stage in neurodevelopment and neurodegenerative processes. Neuroscience 78: 309-324. doi:10.1016/S0306-4522(96)00577-5. PubMed: 9145789.914578910.1016/s0306-4522(96)00577-5

[11] BallatoreC, LeeVM, TrojanowskiJQ (2007) Tau-mediated neurodegeneration in Alzheimer’s disease and related disorders. Nat Rev Neurosci 8: 663-672. doi:10.1038/nrn2194. PubMed: 17684513.1768451310.1038/nrn2194

[12] MuntanéG, DalfóE, MartinezA, FerrerI (2008) Phosphorylation of tau and alpha-synuclein in synaptic-enriched fractions of the frontal cortex in Alzheimer’s disease, and in Parkinson’s disease and related alpha-synucleinopathies. Neuroscience 152: 913-923. doi:10.1016/j.neuroscience.2008.01.030. PubMed: 18343584.1834358410.1016/j.neuroscience.2008.01.030

[13] WillsJ, JonesJ, HaggertyT, DukaV, JoyceJN (2010) Elevated tauopathy and alpha-synuclein pathology in postmortem Parkinson’s disease brains with and without dementia. Exp Neurol 225: 210-218. doi:10.1016/j.expneurol.2010.06.017. PubMed: 20599975.2059997510.1016/j.expneurol.2010.06.017PMC2922478

[14] KaulT, CredleJ, HaggertyT, OaksAW, MasliahE et al. (2011) Region-specific tauopathic changes in brain of the alpha-synuclein overexpressing mouse model of Parkinson’s disease. BMC Neurosci 12:79.2181296710.1186/1471-2202-12-79PMC3176190

[15] DukaT, RusnakM, DroletRE, DukaV, WersingerC et al. (2006) Alpha-synuclein induces hyperphosphorylation of Tau in the MPTP model of parkinsonism. FASEB J 20: 2302-2312. doi:10.1096/fj.06-6092com. PubMed: 17077307.1707730710.1096/fj.06-6092com

[16] DukaT, SidhuA (2006) The neurotoxin, MPP+, induces hyperphosphorylation of Tau in the presence of alpha-Synuclein in SH-SY5Y neuroblastoma cells. Neurotox Res 10: 1-10. doi:10.1007/BF03033329. PubMed: 17000465.1700046510.1007/BF03033329

[17] DukaT, DukaV, JoyceJN, SidhuA (2009) Alpha-Synuclein contributes to GSK-3beta-catalyzed Tau phosphorylation in Parkinson’s disease models. FASEB J 23: 2820-2830. doi:10.1096/fj.08-120410. PubMed: 19369384.1936938410.1096/fj.08-120410PMC2796901

[18] KozikowskiAP, GaisinaIN, PetukhovPA, SridharJ, KingLT et al. (2006) Highly potent and specific GSK-3beta inhibitors that block tau phosphorylation and decrease alpha-synuclein protein expression in a cellular model of Parkinson’s disease. Chemmedchem 1: 256-266. doi:10.1002/cmdc.200500039. PubMed: 16892358.1689235810.1002/cmdc.200500039

[19] HaggertyT, CredleJ, RodriguezO, WillsJ, OaksAW et al. (2011) Hyperphosphorylated Tau in an alpha-synuclein-overexpressing transgenic model of Parkinson’s. Eur J Neurosci: 1-13.10.1111/j.1460-9568.2011.07660.xPMC308695121453448

[20] WillsJ, CredleJ, HaggertyT, LeeJH, OaksAW et al. (2011) Tauopathic changes in the striatum of A53T α-synuclein mutant mouse model of Parkinson’s disease. PLOS ONE 6(3): e17953. doi:10.1371/journal.pone.0017953. PubMed: 21445308.2144530810.1371/journal.pone.0017953PMC3061878

[21] WillsJ, CredleJ, OaksAW, DukaV, LeeJH et al (2012) Paraquat, but not maneb, induces synucleinopathy and tauopathy in striata of mice through inhibition of proteasomal and autophagic pathways. PLOS ONE. 7(1): e30745. doi:10.1371/journal.pone.0030745. PubMed: 22292029. Epub 2012 Jan 23 PubMed: 22292029.2229202910.1371/journal.pone.0030745PMC3264632

[22] PapapetropoulosS, LiebermanA, GonzalezJ, MashDC (2005) Can Alzheimer’s type pathology influence the clinical phenotype of Parkinson’s disease? Acta Neurol Scand 111(6): 353–359. doi:10.1111/j.1600-0404.2005.00411.x. PubMed: 15876335.1587633510.1111/j.1600-0404.2005.00411.x

[23] CrewsL, SpencerB, DesplatsP, PatrickC, PaulinoA et al. (2010) Selective molecular alterations in the autophagy pathway in patients with Lewy body disease and models of alpha-synucleinopathy. PLOS ONE 5(2): e9313. doi:10.1371/journal.pone.0009313. PubMed: 20174468.2017446810.1371/journal.pone.0009313PMC2824828

[24] BueeL, BussiereT, Buee-ScherrerV, DelacourteA, HofPR (2000) Tau proteinisoforms, phosphorylation and role in neurodegenerative disorders. Brain Res Brain Res Rev 33: 95-130.1096735510.1016/s0165-0173(00)00019-9

[25] HashimotoM, RockensteinE, ManteM, MalloryM, MasliahE (2001) beta-Synuclein inhibits alpha-synuclein aggregation: a possible role as an anti-parkinsonian factor. Neuron. 32(2): 213-223. doi:10.1016/S0896-6273(01)00462-7. PubMed: 11683992.1168399210.1016/s0896-6273(01)00462-7

[26] HashimotoM, Bar-OnP, HoG, TakenouchiT, RockensteinE et al. (2004) Beta-synuclein regulates Akt activity in neuronal cells A possible mechanism for neuroprotection in Parkinson’s disease. J Biol Chem 279(22): 23622-9.38.1502641310.1074/jbc.M313784200

[27] NinkinaN, PetersO, MillershipS, SalemH, van der PuttenH et al. (2009) Gamma-synucleinopathy: neurodegeneration associated with overexpression of mouse protein. Hum Mol Genet 18(10): 1779-1794. doi:10.1093/hmg/ddp090. PubMed: 19246516.1924651610.1093/hmg/ddp090PMC2671987

[28] SmithPD, CrockerSJ, Jackson-LewisV, Jordan-SciuttoKL, HayleyS et al. (2003) Cyclin-dependent kinase 5 is a mediator of dopaminergic neuron loss in a mouse model of Parkinson’s disease. Proc Natl Acad Sci U S A 100: 13650-13655. doi:10.1073/pnas.2232515100. PubMed: 14595022. doi:10.1073/pnas.2232515100 PubMed: 14595022 1459502210.1073/pnas.2232515100PMC263868

[29] JensenPH, HagerH, NielsenMS, HojrupP, GliemannJ et al. (1999) alpha-synuclein binds to Tau and stimulates the protein kinase A-catalyzed tau phosphorylation of serine residues 262 and 356. J Biol Chem 274: 25481-25489. doi:10.1074/jbc.274.36.25481. PubMed: 10464279.1046427910.1074/jbc.274.36.25481

[30] QureshiHY, PaudelHK (2011) Parkinsonian neurotoxin 1-methyl-4-phenyl-1,2,3,6-tetrahydropyridine [MPTP] and alpha-synuclein mutations promote Tau protein phosphorylation at Ser262 and destabilize microtubule cytoskeleton in vitro. J Biol Chem 286: 5055-5068. doi:10.1074/jbc.M110.178905. PubMed: 21127069.2112706910.1074/jbc.M110.178905PMC3037617

[31] ForlenzaOV, DinizBS, RadanovicM, SantosFS, TalibLL et al. (2011) Disease-modifying properties of long-term lithium treatment for amnestic mild cognitive impairment: randomised controlled trial. Br J Psychiatry 198(5): 351-356. doi:10.1192/bjp.bp.110.080044. PubMed: 21525519.2152551910.1192/bjp.bp.110.080044

[32] ZhuX, LeeHG, RainaAK, PerryG, SmithMA (2002) The role of mitogen-activated protein kinase pathways in Alzheimer’s disease. Neurosignals 11: 270-281. doi:10.1159/000067426. PubMed: 12566928.1256692810.1159/000067426

[33] KinsS, KurosinskiP, NitschRM, GötzJ (2003) Activation of the ERK and JNK signaling pathways caused by neuron-specific inhibition of PP2A in transgenic mice. Am J Pathol 163(3): 833-843. doi:10.1016/S0002-9440(10)63444-X. PubMed: 12937125.1293712510.1016/S0002-9440(10)63444-XPMC1868255

[34] EcheverriaV, DucatenzeilerA, DowdE, JänneJ, GrantSM et al. (2004) Altered mitogen-activated protein kinase signaling, tau hyperphosphorylation and mild spatial learning dysfunction in transgenic rats expressing the beta-amyloid peptide intracellularly in hippocampal and cortical neurons. Neuroscience 129: 583-592. doi:10.1016/j.neuroscience.2004.07.036. PubMed: 15541880.1554188010.1016/j.neuroscience.2004.07.036

[35] AndoK, UemuraK, KuzuyaA, MaesakoM, Asada-UtsugiM et al. (2011) N-cadherin regulates p38 MAPK signaling via association with JNK-associated leucine zipper protein: implications for neurodegeneration in Alzheimer disease. J Biol Chem 286: 7619-7628. doi:10.1074/jbc.M110.158477. PubMed: 21177868.2117786810.1074/jbc.M110.158477PMC3045016

[36] HangerDP, BettsJC, LovinyTL, BlackstockWP, AndertonBH (1998) New phosphorylation sites identified in hyperphosphorylated tau [paired helical filament-tau] from Alzheimer’s disease brain using nanoelectrospray mass spectrometry. J Neurochem 71: 2465-2476. PubMed: 9832145.983214510.1046/j.1471-4159.1998.71062465.x

[37] TroquierL, CaillierezR, BurnoufS, Fernandez-GomezFJ, GrosjeanME et al. (2012) Targeting phospho-Ser422 by active Tau Immunotherapy in the THYTau22 mouse model: a suitable therapeutic approach . Curr Alzheimer Res 9(4): 397-405. doi:10.2174/156720512800492503. PubMed: 22272619.2227261910.2174/156720512800492503PMC3637173

